# Comprehensive Analysis of the Expression and Prognosis for E2Fs in Human Clear Cell Renal Cell Carcinoma

This article has been retracted.

**DOI:** 10.1155/2021/5790416

**Published:** 2021-09-06

**Authors:** Chongli Zhang, Yong Cui, Guannan Wang, Wugan Zhao, Haiyu Zhao, Xuejie Huang, Min Zhang, Wencai Li

**Affiliations:** ^1^Department of Pathology, The First Affiliated Hospital of Zhengzhou University, Zhengzhou, China; ^2^Department of Pathology, School of Basic Medical Sciences, Zhengzhou University, Zhengzhou, China; ^3^Department of Urology, The First Affliated Hospital of Henan University of CM, Zhengzhou, China; ^4^Department of Pathology, Zhengzhou Central Hospital, Zhengzhou, China

## Abstract

**Background:**

E2F transcription factors is a family of transcription factors, and lots of studies have shown that they play a key role in the occurrence and development of many tumors. However, the association between expression, prognostic value, and immune infiltration in the tumor microenvironment of the eight E2Fs members in ccRCC is still unclear.

**Method:**

s. We used online databases, such as ONCOMINE, UALCAN, Kaplan–Meier plotter, GEPIA, Metascape, TIMER, and cBioPortal, to analyze the effect of mRNA expression of E2Fs family members in ccRCC on the prognosis of patients and the relationship with immune infiltration.

**Results:**

Except for E2F5, other seven members of the family of E2Fs mRNA expression levels in ccRCC tissues were significantly higher than control tissues. And the high expression of E2Fs mRNA in ccRCC patients was related to cancer stage and tumor grade. Survival analysis results suggested that elevated mRNA expression levels of E2F1/2/3/4/7/8 were significantly related to the shorter overall survival (OS) in ccRCC patients (*P* = 3.9*E* – 06), while high mRNA expression of E2F6 is not related to OS (*P* = 0.061). Mutations of E2Fs were correlated with shorter OS of ccRCC patients (*P* = 7.094*E* – 5). In addition, mRNA expression of E2F1/2/3/4/7/8 was positively correlated with infiltration of six types of immune cells, including B cells, CD8+ T cells, CD4+ T cells, macrophages, neutrophils, and dendritic cells.

**Conclusions:**

These results indicate that E2F1/2/3/4/7/8 may be used as a prognostic marker for the survival of ccRCC patients and laid the foundation for studying the immune infiltration role of E2Fs family members in tumors.

## 1. Introduction

Renal cell carcinoma (RCC) is a malignant tumor originating from the kidney parenchyma, referred to as kidney cancer. According to the 2016 WHO Classification of Renal Tumors, renal cell tumors are divided into 16 subtypes such as renal clear cell carcinoma and tubular cystic renal cell carcinoma [1]. Clear cell renal cell carcinoma (ccRCC) is the most common pathological type of RCC and has a poor prognosis, accounting for 75%–80% of RCC, and is also the most aggressive [2]. Surgery is the main treatment for patients with CC RCC at present; while traditional radiotherapy and chemotherapy have certain tolerance to CC RCC, especially for advanced or metastatic CC RCC patients, there is still a lack of effective treatment [3]. Therefore, research and prediction of biomarkers and therapeutic targets that are meaningful to ccRCC patients are particularly important for the survival and prognosis of ccRCC patients.

The E2F transcription factors family was first studied in the 1980s and was initially identified as an activator of the E2 gene promoter of adenovirus [4]. Sequence-based homology and function, eight different members of the E2Fs transcription factor (E2F1–E2F8) have been identified to date. Studies have found that E2Fs play an important role in transcription, apoptosis, and tumor occurrence and inhibition. Various factors can interact and influence each other [5–7]. E2Fs can form complexes with retinoblastoma protein (RB) proteins, including RB, P107, and P130, which jointly regulate gene expression [8]. Mutations in genes often lead to the loss of RB protein function, which leads to the overactivation of E2Fs, thus deregulating cell proliferation.

Previous studies have found that some E2Fs family members mRNA were abnormally expressed in ccRCC patients and had a negative impact on the prognosis of patients [9, 10]. However, the role of different E2Fs family members in the genesis and development of ccRCC remains unknown. In this study, analyzing the expression differences, mutations, and prognostic significance of different E2Fs mRNA in ccRCC patients based on multiple large databases may help to further understand its potential roles in ccRCC.

## 2. Materials and Methods

### 2.1. ONCOMINE Database Analysis

ONCOMINE database (http://.oncomine.org) is an open database and integrated data mining platform based on gene chips, which helps to promote the research of whole genome expression analysis. In this database, you can set the conditions for screening and mining data according to your own needs [11]. In this study, ONCOMINE was used to analyze the mRNA levels of E2F family members in ccRCC, and difference of transcriptional expression was contrasted by Student's *t*-test. Enter relevant filter conditions in the data retrieval interface: *P* value = 0.01; fold change = 1.5; gene rank = 10%; and data type: mRNA. A comparative analysis of cancer specimens and normal control data sets was performed for each gene.

### 2.2. UALCAN Database Analysis

UALCAN (http://ualcan.path.uab.edu) is an effective online analysis website for cancer data. It is mainly used for in-depth analysis of gene expression data of 31 types of cancer in the TCGA project. This database can classify tumors by stage and race or other clinicopathological characteristics as the basis; divide various tumors into different subgroups, and estimate the impact of gene expression levels and clinicopathological characteristics on patient survival [12]. Difference of transcriptional expression was compared by Student's *t*-test. Here, we used UALCAN to analyze the relationship between the mRNA expression of 8 E2Fs family members in primary ccRCC tissues and clinicopathological characteristics.

### 2.3. Kaplan–Meier Plotter

Kaplan–Meier plotter (http://kmplot.com/analysis) can be used to evaluate the impact of mRNA, micRNA, and protein on the survival of 21 cancers, including bladder cancer, pancreatic cancer, liver cancer, breast cancer, ovarian cancer, lung cancer, gastric cancer, etc. [13–18]. The sources of the database include Gene Expression Omnibus (GEO), European Genome-Phenome Archive (EGA), and The Cancer Genome Atlas (TCGA). This study includes gene expression data and survival information of 530 ccRCC patients. The main purpose of this study was to discover and verify survival biomarkers based on meta-analysis. In Kaplan–Meier plotter, patients were divided into two groups with high and low expression according to the median value of mRNA expression, and the number at risk cases is verified by the KM survival curve. The number of at-risk cases, the median value of mRNA expression, HR, 95% CI, and *P* value were shown in the Kaplan–Meier plotter verification page. When *P* value was <0.05, the difference was considered statistically significant.

### 2.4. TCGA and cBioPortal Analysis

The Cancer Genome Atlas (TCGA) database is currently the largest tumor gene information database, containing high-throughput sequencing of more than 30 cancers, gene methylation, copy number changes, point mutations, and other data. A large number of cancer gene maps can be systematically analyzed to find out gene variations in the process of tumor genesis and understand the pathological mechanisms of tumor genesis and development [19]. cBioPortal (http://.cbioportal.org) is an online, open resource for exploring, visualizing, and analyzing multidimensional cancer genome data [20]. In this research, 510 ccRCC samples from the TCGA database were obtained from cBioPortal database. We analyzed the genomic information of 8 E2Fs family members using the database filtering option, which contained mutations, putative copy-number alterations from GISTIC, and mRNA Expression *z*-Scores (RNASeq V2 RSEM) with a *z*-score threshold of 1.8. According to cBioPortal online guidance to obtain E2Fs member gene mutations and ccRCC patients with OS and DFS plotter. *P* value <0.05 is considered to indicate statistical significance.

### 2.5. Analysis of GEPIA Data Sets

The Online Database Gene Expression Profiling Interactive Analysis (GEPIA) (http://gepia.cancer-pku.cn/index.html) is a newly developed interactive web server for analyzing the RNA sequencing expression data of 9,736 tumors and 8,587 normal samples from the TCGA and the GTEx projects, such as tumor/normal differential expression analysis, profiling according to cancer types or pathological stages, patient survival analysis, similar gene detection, and correlation analysis [21]. We used the GEPIA2 module of the GEPIA database to obtain 160 coding genes in ccRCC with similar functions to 8 members of the E2Fs family.

### 2.6. Analysis of Metascape Data Sets

Metascape (http://metascape.org) is a portal site that provides gene annotation and enrichment analysis, provides automated meta-analysis tools, supports BioGrid-based protein-protein interaction analysis, namely, PPI analysis, and supports gene-based Theory (GO) network interactive visualization and KEGG pathway enrichment [22]. We used Metascape to perform gene ontology (GO) classification and KEGG pathway enrichment analysis on 160 similar genes of E2Fs family members. Parameter setting: *P* value < 0.05, min enrichment > 3, and min overlap > 3 were considered as significant.

### 2.7. Analysis of TIMER Data Sets

Tumor IMmune Estimation Resource (TIMER) (https://cistrome.shinyapps.io/timer/) is a web server for comprehensive analysis of tumor-infiltrating immune cells. The abundances of six immune infiltrates (B cells, CD4+ T cells, CD8+ T cells, neutrophils, macrophages, and dendritic cells) were estimated by TIMER algorithm [23]. The correlation between E2F1/2/3/4/7/8 expression in ccRCC and infiltration level of immune cells was analyzed by gene module in TIMER database.

## 3. Results

### 3.1. Overexpression of Different E2Fs Family Members mRNA in ccRCC Patients

The transcriptional levels of mRNA in 8 E2Fs family members from 20 cancers were compared with normal tissue samples using the ONCOMINE database (Figure 1 and Table 1). As shown in Figure 1, E2F1/3/4 mRNA overexpression was found in ccRCC patients in multiple data sets. Only a significant increase in the transcription level of E2F3 was found in the mRNA expression data set of ccRCC patients, in the Jones Renal data set, the fold change was 1.575, and the *P* value was 7.97E-05. E2F1 mRNA expression has no significant difference (fold change <1.5, *P* value >0.05). Although the transcription level of E2F4 was slightly higher than that of normal kidney tissue, the *P* value did not exceed 0.05, but the fold change was <1.5.

This figure showed the number of statistically significant data sets where target gene mRNA was overexpressed or downregulated (red: overexpression; blue: downregulation). Cut-off of *P* value and fold change were as follows: *P* value: 0.01, fold change: 1.5, gene rank: 10%, and data type: mRNA.

### 3.2. Relationship between Different E2Fs mRNA Expression Levels and Clinicopathological Parameters in Patients with ccRCC

We analyzed the level of mRNA expression in different E2Fs family members of ccRCC patients and normal renal tissues using UALCAN database (Figure 2). The results showed that the expression of E2F1/2/3/4/6/7/8 mRNA in ccRCC tissues was significantly higher than that in normal tissues (*P* < 0.05), while the expression of E2F5 mRNA in normal tissues was not significantly higher than that in tumor tissues. Then, correlation between the mRNA expression of E2Fs family members was analyzed in ccRCC patients and cancer stage (Figure 3) and tumor grade (Figure 4). As shown in Figure 3, apart from E2F5, the high expression of E2F1/2/3/4/6/7/8 member mRNA in tumor tissues was correlated with the cancer stage of the patients, and the E2F1/2/7/8 mRNA expression level was at stage IV highest. The data in Figure 4 showed that the high expression of E2F1/2/3/4/6/7/8 member mRNA in tumor tissues was correlated with the patient's tumor grade, and the level of E2F1/2/3/7/8 mRNA expression was also the highest in grade IV. These results indicated that mRNA expression of seven E2Fs family members was correlated with cancer stage and tumor grade in ccRCC patients, except for E2F5.

### 3.3. Prognostic Value of E2Fs mRNA Expression in ccRCC Patients

Next, we further analyzed the relationship between the mRNA expression of different E2Fs family members in ccRCC patients and the prognosis of ccRCC patients using Kaplan–Meier plotter (http://kmplot.com/analysis/). As shown in Figure 5, the relationship between the members with high mRNA expression of the E2Fs family members and the prognosis of ccRCC patients was first combined and analyzed (Figure 5(a)). The combined analysis results showed that in ccRCC patients, E2Fs members with high mRNA expression were associated with poor OS (HR = 1.99, 95% CI: 1.48–2.69, *P* = 3.9*E* − 06). Then, we separately studied the relationship between the mRNA expression level of each member of the E2Fs family and the prognosis of ccRCC patients (Figures 5(b)–5(i)). The high mRNA expression of E2F1 (HR = 2.01, 95％CI: 1.48–2.73, *P* = 4.6*E* − 06), E2F2 (HR = 2.16, 95％CI: 1.89–3.85, *P* = 1.3*E* − 05), E2F3 (HR = 1.66, 95％CI: 1.21–2.28, *P* = 0.0014), E2F4 (HR = 1.86, 95％CI: 1.37–2.52, *P*= 5*E* − 05), E2F5 (HR = 2.14, 95％CI: 1.57–2.92, *P* = 4.6*E* − 06), E2F7 (HR = 2.22, 95％CI: 1.63–3.02, *P* = 2.2*E* − 07), and E2F8 (HR = 1.62, 95％CI: 1.22–2.22, *P* = 0.00091) were significantly correlated with shorter OS in ccRCC patients, but no statistically significant association was found between E2F6 mRNA expression and OS (HR = 1.4, 95% CI: 0.98–1.98, *P* = 0.061). These results indicated that the mRNA expression of E2F1/2/3/4/5/7/8 was significantly related to the prognosis of ccRCC patients, and they may be used as biomarkers to predict survival in patients with ccRCC.

### 3.4. Gene Mutation of E2Fs in ccRCC Patients and Its Association with OS and Disease-Free Survival (DFS)

cBioPortal was used to analyze the genetic variation of E2Fs family members and its effect on OS and DFS in patients with ccRCC. As shown in Figure 6(a), sequence changes in E2Fs occurred in 142 (28%) of 510 ccRCC patients. Apart from E2F8, all the other 7 E2Fs mutations rates exceeded 5%. The mutation rate of E2F1 was the highest (8%). The mutation rates of E2F4, E2F6, E2F3, E2F7, E2F2, and E2F5 were 7%, 7%, 6%, 6%, 5%, and 5%, respectively. The results of Kaplan–Meier plotter and log-rank test indicated that the genetic change of E2Fs was correlated with shorter OS of ccRCC patients (Figure 6(b), *P* = 7.094*E* − 5), but the genetic change of E2Fs was not correlated with DFS in ccRCC patients (Figure 6(c), *P* = 0.110).

### 3.5. Enrichment Analysis of Similar Functional Genes of E2Fs Members in ccRCC Patients

Enrichment analysis is helpful for us to further understand the biological functions of the E2Fs family in ccRCC. First, through the similar genes detection module in GEPIA2, 160 coding genes with similar functions to E2F1-E2F8 are obtained. Then, we used the Metascape database to perform GO and KEGG enrichment analysis on these 160 coding genes. The top 20 GO analysis consists of three parts: biological processes (11 items), cellular components (7 items), and molecular function (2 items) (Figures 7(a) and 7(b) and Table 2). The terms of biological process mainly included GO : 0051301 (cell division), GO : 0010564 (regulation of cell cycle process), GO : 0006260 (DNA replication), GO : 0007080 (mitotic metaphase plate congression), and GO : 0071103 (DNA conformation change); the terms of cellular component mainly included GO : 0005819 (spindle), GO : 0005815 (microtubule organizing center), GO : 1990234 (transferase complex), and GO : 0031261 (DNA replication preinitiation complex); and the terms of molecular function mainly included GO : 0043021 (ribonucleoprotein complex binding) and GO : 0003682 (chromatin binding).

As shown in Figures 7(c) and 7(d) and Table 3, there were seven KEGG pathways that were significantly associated with E2Fs similar genes in ccRCC : ko04110 (cell cycle), ko03460 (Fanconi anemia pathway), ko05168 (herpes simplex infection), ko04115 (p53 signaling pathway), hsa03040 (spliceosome), ko00310 (lysine degradation), and hsa05161 (hepatitis B).

### 3.6. Correlation between mRNA Expression of E2Fs Family Members and Immune Infiltration Level in ccRCC Patients

Combined with the above analysis results of the E2Fs family in ccRCC patients, we analyzed the correlation between the six transcription factors E2F1/2/3/4/7/8 and tumor immune cells in ccRCC patients and found that these six transcription factors were significantly negatively correlated with tumor purity in ccRCC patients. E2F2 expression was significantly positively correlated with B cell (*r* = 0.401, *P* = 3.66*e* − 19), CD8+ T cell (*r* = 0.296, *P* = 2.76*e* − 10), CD4+ T cell (*r* = 0.345, *P*= 2.71*e* − 14), macrophage (*r* = 0.298, *P* = 1.28*e* − 10), neutrophil (*r* = 0.458, *P* = 4.49*e* − 25), and dendritic cell (*r* = 0.345, *P* = 2.71*e* − 14) (Figure 8(b)). Similarly, E2F3 expression was also positively correlated with B cell (*r* = 0.345, *P* = 3.00*e* − 10), CD8+ T cell (*r* = 0.282, *P* = 1.88*e* − 9), CD4+ T cell (*r* = 0.339, *P* = 8.21*e* − 14), macrophage (*r* = 0.451, *P*= 7.27*e* – 24), neutrophil (*r* = 0.534, *P* = 3.92*e* − 35), and dendritic cell (*r* = 0.452, *P* = 2.46*e* − 24) (Figure 8(c)). E2F1 expression was positively correlated with B cell (*r* = 0.122, *P* = 9.05*e* − 03), CD4+ T cell (*r* = 0.159, *P* = 6.04*e* − 04), macrophage (*r* = 0.093, *P* = 4.94*e* − 02), neutrophil (*r* = 0.161, *P* = 5.22*e* − 04), and dendritic cell (*r* = 0.192, *P* = 3.90*e* − 05) (Figure 8(a)) immune infiltration. The expression of E2F4/7/8 was correlated with all the six immune cells, especially the expression of E2F4 was associated with CD4+ T cell (*r* = 0.356, *P* = 3.58*e* − 15) and neutrophil (*r* = 0.359, *P* = 2.09*e* − 15) (Figure 8(d)); E2F7 expression and B cell (*r* = 0.284, *P* = 5.56*e* − 10), neutrophil (*r* = 0.435, *P* = 1.30*e* − 22), dendritic cell (*r* = 0.37, *P* = 3.32*e* − 16) (Figure 8(e)). Immune infiltration is significantly positively correlated; the same as E2F7, E2F8 expression is related to B cell (*r* = 0.312, *P* = 8.70*e* − 12), macrophage (*r* = 0.306, *P* = 3.68*e* − 11), neutrophil (*r*= 0.317, *P* = 3.58*e* − 12), dendritic cell (*r* = 0.354, *P* = 7.35*e* − 15) (Figure 8(f)) immune infiltration also showed a significant positive correlation. The above results indicated that the E2Fs family may be involved in the immune infiltration process of ccRCC cells.

## 4. Discussion

So far, lots of literatures have reported that abnormal expression of E2Fs family gene plays an important role in the development of cancers, including gastric cancer, ovarian cancer, liver cancer, and colon cancer [28–31]. Some members of E2Fs have also been reported to play a key role in renal clear cell carcinoma [32], but the different roles of E2Fs family members in ccRCC remain to be clarified. In this study, we attempted to systematically analyze the expression levels, mutations, and prognostic value of different E2Fs family members in renal clear cell carcinoma.

E2F1 transcription factor is well known as cell cycle regulator and as an effective mediator of DNA damage-induced apoptosis and checkpoint response. Understanding the diversity of E2F1 activity and its seemingly dichotomous function has been a focus of research. Although the E2Fs pathway is often deregulated in cancer, the roles of E2F1 as a proliferation or cell death promoter in tumorigenesis are still far from being understood [33, 34]. Numerous studies indicate that E2F1 transcription factor is one of the most in-depth E2Fs family members in tumor research, and the high expression of E2F1 is of great significance for the poor prognosis of malignant tumors such as gastric cancer [35], hepatocellular carcinoma [36], pancreatic cancer [37], and prostate cancer [38]. Ma et al. [9] have first reported that the mRNA level of E2F1 in renal clear cell carcinoma tissue is related to tumor pathological parameters, including diameter, Fuhrman tumor grade, pT staging, TNM staging and macrovascular infiltration (MAVI), and E2F1 expression with the increase of tumor tissue grade; they also found that E2F1 has promoting effects on the proliferation, migration, and invasion of cancer cells. Similar to our research, high expression of E2F1 mRNA was significantly associated with tumor staging and poor survival in ccRCC and was an independent prognostic factor for shorter OS in ccRCC.

E2F2 is a transcriptional activator. Although E2F2 has not been studied as carefully as E2F1, it plays a key role in many cellular processes such as cell cycle regulation, proliferation, differentiation, and cancer development [39–41]. Gao et al. [42] have found that compared with the normal tissues, the miR-155 activity in ccRCC tissues is significantly upregulated. miR-155 can downregulate the expression of E2F2 by directly binding to the 3′-UTR of E2F2, thus inhibiting the migration and invasion of ccRCC cells. Our analyses found that the expression levels of mRNA and protein of E2F2 in ccRCC tissues were significantly higher, and the expression of E2F2 was significantly related to the tumor stage and poor survival rate of ccRCC patients. These indicated that E2F2 might play an active role in the occurrence and development of renal clear cell carcinoma.

E2F3 is also a member of the E2Fs family, and two subtypes of E2F3a and E2F3b have been found. E2F3a is mainly expressed in S phase, while E2F3b is active in the whole cell cycle. Studies have reported that the activity of E2F3 acute loss affects the coding DNA replication and mitotic activity of gene expression, the loss of E2F1 can influence a limited number of genes that are distinct from those regulated by E2F3, the activity of E2Fs long-term loss leads to the compensation of the other members, and acute function loss analysis reveals the special roles of these proteins [43]. Gao et al. [10] have determined that HIF-2*α* is the direct target gene upregulated by E2F3 in vitro cell experiments and the construction of mouse tumor models. However, some scholars have pointed out that the relative expression level of E2F3 mRNA in tumor tissues is lower than that in adjacent tissues, and the downregulation of E2F3 expression may play a role in the formation of ccRCC and may promote the malignant progression of cancer [44]. In our study, E2F3 expression in ccRCC was higher than that in normal tissues and was significantly negatively correlated with cancer stage and tumor pathological grade. In addition, high expression of E2F3 was significantly associated with poor OS in patients with renal clear cell carcinoma.

E2F4 is originally identified as a transcriptional suppressor whose activity is essential for participating in and maintaining cell cycle arrest in G0/G1 with members of the retinoblastoma (RB). Hsu et al. [45] recently have found that E2F4 not only has cell cycle regulation effect, but also has effects on the regeneration process of embryonic and adult stem cells and the occurrence and development of cancer. Furthermore, E2F4 can directly activate the target genes, and this process is independent of the RB family. Kim et al. [46] have shown that higher E2F4 expression in renal clear cell carcinoma samples than normal kidney samples, and high E2F4 expression is not correlated with OS and PFS in ccRCC patients. In our study, E2F4 was significantly overexpressed in ccRCC tissues compared to normal, and our results first suggested that high E2F4 mRNA expression was significantly related to the cancer stage and tumor grade of ccRCC patients, and high E2F4 mRNA expression was related to poor OS in ccRCC patients.

Studies have shown that abnormal expression of E2F5 is associated with a variety of tumors, such as esophageal squamous cell carcinoma and hepatocellular carcinoma [47, 48]. Jiang et al. have reported for the first time that E2F5 is usually overexpressed in primary liver cancer, while E2F5 knockdown significantly inhibits the growth of liver cancer cells. Similarly, Ishimoto et al. have found that the high expression of E2F5 in esophageal squamous cell carcinoma may be related to the poor prognosis of ESCC patients. In this study, we found that the mRNA expression of E2F5 in normal kidney tissue was higher than ccRCC tissue. However, OS showed the high expression of E2F5 was significantly related to the poor survival rate of ccRCC patients. We guessed that the reason for this result was the sample size is too small, and the exact roles of E2F5 in ccRCC need further evaluation.

Transcription factor E2F6 is known to be abnormally expressed in many malignancies, including gastric cancer and breast cancer [49, 50]. However, the expression pattern and prognosis of E2F6 mRNA in ccRCC remain unclear. In this study, we reported that E2F6 mRNA expression in ccRCC tissues was higher than that in normal kidney tissues, but E2F6 was not associated with OS in ccRCC patients.

E2F7, a newly discovered member of the family of atypical E2Fs transcription factors, has two unique DNA binding domains and lacks typical Rb egg self-binding domain [51, 52]. Studies have shown that abnormal expression of E2F7 in a variety of malignant tumors may be involved in the occurrence and development of tumors, such as skin squamous cell carcinoma, endometrial carcinoma, etc. [53, 54]. Yin et al. [55] have found that E2F7 may be a prognostic factor affecting the survival of glioma patients and is a promising potential target for the treatment of this disease. So far, no literature has reported the roles of E2F7 in ccRCC. In this study, it was found that the expression of E2F7 mRNA in ccRCC tissues was significantly higher than that in normal tissues, and the expression of E2F7 in ccRCC patients was significantly correlated with cancer stage and tumor pathology. In addition, in ccRCC patients, the high expression of E2F7 was significantly correlated with relatively poor survival, suggesting that E2F7 plays a carcinogenic role in ccRCC.

As a newly discovered member, E2F8 has the characteristics of repeated DNA binding domains that are different from E2F1-E2F6 and regulates gene expression in a dimer-independent manner. Its function is not fully understood and E2F8 is known to play an important role in embryonic development and cell cycle control by inhibiting E2F1 [56, 57]. Kim et al. [58] have shown that E2F8 is highly correlated with PFS in cervical cancer patients. Park et al. [59] have pointed out that E2F8 is overexpressed in lung cancer and is necessary for the growth of lung cancer cells, suggesting that E2F8 might be a novel therapeutic target for lung cancer treatment. Similar to E2F7, this study found that the mRNA expression of E2F8 was significantly increased in ccRCC tissue for the first time. The mRNA expression of E2F8 was significantly related to the cancer stage and tumor grade of patients with ccRCC, and the high expression of E2F8 mRNA was significantly related to the shorter OS of ccRCC patients. It may function as an independent prognostic factor for shorter OS in ccRCC patients. The above results indicate that E2F8 plays a carcinogenic effect in ccRCC.

Our analysis of the genetic variation of a single gene of E2Fs family members found that the percentage of genetic variation of a single gene was related to the shorter OS but not related to DFS. By constructing coding genes with similar functions in the E2Fs family to perform GO and KEGG enrichment analysis charts, it is helpful to accurately understand the biological processes and related pathways that E2Fs participating in ccRCC. The results showed that these genes were mainly involved in cell division, cell cycle regulation, and P53 signaling pathway.

Tumor-infiltrating immune cells are an important part of the tumor microenvironment. Studies have shown that tumor-infiltrating immune cells can secrete growth factors [60], inhibit cell apoptosis [61], promote angiogenesis, and promote tumor growth and metastasis [62], and the current tumor immune microenvironment has become an important therapeutic target. Our studies displayed that the mRNA expression level of E2F1/2/3/4/7/8 was positively correlated with the level of immune cells infiltration, including B cells, CD8+ T cells, macrophages, neutrophils, and dendritic cells. It suggested that these transcription factors might be involved in the immune infiltration process of ccRCC cells, which provided a new research direction for the treatment of ccRCC.

Although our research has provided various evidences for E2Fs family members as molecular markers of ccRCC, further studies on their detailed mechanism of action are needed to promote E2Fs as diagnostic markers or therapeutic targets for ccRCC.

## 5. Conclusions

In summary, we studied the expression, mutation, and prognostic value of different E2Fs members in ccRCC patients with professional and reliable statistical data analysis system. Except for E2F5, the mRNA overexpression of E2Fs members was correlated with the clinical cancer stage and tumor pathological grade of ccRCC patients. In addition, high mRNA expression of E2F1/2/3/4/7/8 was significantly associated with poorer OS in ccRCC patients, and also positively correlated with the level of tumor immune cell infiltration. It was also observed that genetic changes (28%) of E2Fs in ccRCC patients were associated with shorter OS. These results indicate that E2F1/2/3/4/7/8 may be a prognostic biomarker for survival in ccRCC patients and may be used as a promising potential target for the treatment of ccRCC.

## Figures and Tables

**Figure 1:** Transcription expression of the E2Fs family in 20 different types of cancer (ONCOMINE database).

**Figure 2:** mRNA expression of different E2Fs family members in ccRCC and adjacent normal renal tissues (UALCAN). mRNA expression of E2Fs family members (E2F1/2/3/4/6/7/8) was overexpressed in primary renal tissue (a–h) compared with normal renal tissue. ^*∗*^*P* < 0.05, ^*∗∗*^*P* < 0.01, and ^*∗∗∗*^*P* < 0.001.

**Figure 3:** The relationship between the mRNA expression of different E2Fs family members in the TCGA database and the cancer stage of ccRCC patients. The mRNA expression of E2Fs family members (E2F1/2/3/4/6/7/8) was correlated with the cancer stage of patients (including data from 72 normal people and 531 ccRCC patients). ^*∗*^*P* < 0.05, ^*∗∗*^*P* < 0.01, and ^*∗∗∗*^*P* < 0.001.

**Figure 4:** The relationship between the mRNA expression of different E2Fs family members in the TCGA database and the tumor pathological grade of ccRCC patients. mRNA expression of E2Fs family members (E2F1/2/3/4/6/7/8) was correlated with tumor pathological grade in patients (including data from 72 healthy subjects and 531 ccRCC patients). ^*∗*^*P* < 0.05, ^*∗∗*^*P* < 0.01, and ^*∗∗∗*^*P* < 0.001.

**Figure 5:** Kaplan–Meier curve revealing the OS difference based on E2F mRNA levels in ccRCC patients (Kaplan–Meier plotter). High mRNA expression of the E2Fs family was associated with poorer OS of patients with ccRCC (a). High mRNA expression in E2F1/2/3/4/5/7/8 was significantly associated with shorter OS of patients with ccRCC (b–f, h, i), while high mRNA expression in E2F6 was not associated with prognosis in patients of ccRCC (g).

**Figure 6:** E2Fs gene mutation and association with OS and DFS in ccRCC patients (cBioPortal). (a) Mutation frequency of E2Fs family members and adjacent genes in ccRCC patients. (b) E2Fs mutation was associated with poor overall survival of ccRCC patients. (c) In ccRCC patients, E2Fs mutation was not associated with DFS.

**Figure 7:** Enrichment analysis of 160 functionally similar genes from 8 E2Fs family members in ccRCC. (a) GO enrichment analysis results. (b) KEGG enrichment analysis results. (c) Network of GO and KEGG enriched terms colored by *P* value, (d) where terms containing more genes tend to have a more significant *P* value.

**Figure 8:** The correlation between the mRNA expression level of E2Fs (E2F1/2/3/4/5/7/8) and the level of immune infiltration in clear cell renal cell carcinoma (TIMER).

**Table 1:** E2Fs transcriptional level between ccRCC and normal renal tissues (ONCOMINE database).

	Types of ccRCC vs. normal	Fold change	*P* value	*t*-test	Reference
E2F1	ccRCC	1.118	0.094	1.376	Yusenko et al. [24]

E2F3	ccRCC	1.575	7.97E-05	4.133	Jones et al. [25]
	ccRCC	1.421	0.011	2.574	Beroukhim et al. [26]

E2F4	ccRCC	1.1	0.056	1.684	Lenburg et al. [27]
	ccRCC	1.11	0.016	2.216	Jones et al. [11]

ccRCC: clear cell renal cell carcinoma. *P* < 0.05 was considered as a significant difference.

**Table 2:** Analysis of GO function enrichment of E2Fs family members and 160 functionally similar genes in ccRCC.

GO	Category	Description	Count	%	Log10 (*P*)	Log10 (*q*)
GO : 0051301	GO biological processes	Cell division	32	22.22	−22.64	−18.29
GO : 0010564	GO biological processes	Regulation of cell cycle process	30	20.83	−17.11	−13.6
GO : 0005819	GO cellular components	Spindle	19	13.19	−13.23	−10.06
GO : 0006260	GO biological processes	DNA replication	17	11.81	−13.12	−10
GO : 0005815	GO cellular components	Microtubule organizing center	21	14.58	−9.18	−6.33
GO : 0007080	GO biological processes	Mitotic metaphase plate congression	7	4.86	−8.17	−5.45
GO : 0071103	GO biological processes	DNA conformation change	13	9.03	−7.83	−5.16
GO : 1990234	GO cellular components	Transferase complex	18	12.50	−7.01	−4.41
GO : 0007062	GO biological processes	Sister chromatid cohesion	6	4.17	−6.05	−3.52
GO : 0031261	GO cellular components	DNA replication preinitiation complex	3	2.08	−5.88	−3.35
GO : 0000076	GO biological processes	DNA replication checkpoint	4	2.78	−5.82	−3.3
GO : 0006513	GO biological processes	Protein monoubiquitination	6	4.17	−5.81	−3.3
GO : 0016363	GO cellular components	Nuclear matrix	7	4.86	−5.80	−3.3
GO : 0030496	GO cellular components	Midbody	8	5.56	−5.31	−2.86
GO : 0043021	GO molecular functions	Ribonucleoprotein complex binding	7	4.86	−5.22	−2.79
GO : 0016607	GO cellular components	Nuclear speck	11	7.64	−5.11	−2.71
GO : 0003682	GO molecular functions	Chromatin binding	13	9.03	−4.87	−2.51
GO : 0016570	GO biological processes	Histone modification	11	7.64	−4.47	−2.2
GO : 0022613	GO biological processes	Ribonucleoprotein complex biogenesis	11	7.64	−4.09	−1.91
GO : 0006368	GO biological processes	Transcription elongation from RNA polymerase II promoter	5	3.47	−4.05	−1.87

**Table 3:** KEGG functional enrichment analysis of E2Fs family members and 160 similar functional genes in ccRCC.

GO	Category	Description	Count	%	Log10 (*P*)	Log10 (*q*)
ko04110	KEGG pathway	Cell cycle	9	6.25	−7.77	−4.93
ko03460	KEGG pathway	Fanconi anemia pathway	4	2.78	−3.76	−1.33
ko05168	KEGG pathway	Herpes simplex infection	6	4.17	−3.40	−1.22
ko04115	KEGG pathway	p53 signaling pathway	4	2.78	−3.35	−1.22
hsa03040	KEGG pathway	Spliceosome	5	3.47	−3.18	−1.18
ko00310	KEGG pathway	Lysine degradation	3	2.08	−2.45	−0.55
hsa05161	KEGG pathway	Hepatitis B	4	2.78	−1.87	−0.08

## Data Availability

All data for this study are sourced from public databases, and the original data can be provided by the corresponding author upon reasonable request.
